# The analysis and solution for intercity travel behaviors during holidays in the post-epidemic era based on big data

**DOI:** 10.1371/journal.pone.0288510

**Published:** 2023-07-19

**Authors:** Xike Zhang, Jiaqi Gao

**Affiliations:** 1 China Academy of Transportation Sciences, Beijing, China; 2 School of Traffic and Transportation, Beijing Jiaotong University, Beijing, China; Shenzhen University, CHINA

## Abstract

The COVID-19 had a huge impact on the transportation industry. In the post-epidemic stage, intercity transportation will face great challenges as places are unsealed, tourism and other service industries begin to recover, and residents’ travel demand gradually increases. An in-depth study of residents’ intercity travel behavior during holidays in the post-epidemic era will help restore public trust in public transportation and improve the quality of public transportation services. Based on traditional research on ways of travelling, the study adopted the Complex Network Analysis Theory. The city clusters of Shandong Peninsula were taken as the research region. The research studied the impact of the differences in regional attributes of the cities in Shandong Peninsula on residents’ intercity travel in the post-epidemic times. A dynamic evolution model of how residents choose to travel was built to simulate the changes to their ways of traveling in the post-epidemic era under two conditions, which are: traveling under the government’s supervision of intercity travel and traveling under the government’s optimization of intercity travel conditions. The conclusions drawn from the analyses of Complex Network Theory and Evolutionary Game Theory are as follows. First, in the holiday intercity travel in the post-epidemic times, the neighboring cities of Shandong Peninsula are closely connected, thus traveling between neighboring cities dominates intercity travel. Second, the travel network concentration of residents on long-term holidays is lower than that on short-term holidays, and the migration intensity of residents is higher than that on short-term holidays, while the willingness of residents’ migration on short-term holidays is higher than that on long-term holidays. The willingness to migrate on holidays is generally lower than that before the epidemic. Third, in a normal intercity travel network, the travel between two cities with medium and long distances is mainly by public transport. However, the dominance of public transport will be affected under the impact of the epidemic. In short-distance travel between two cities, private transport is in an advantageous position, and under the impact of the epidemic, this advantage will become more significant. The government can improve the position of public transport in short-distance travel by making optimizations.

## 1. Introduction

According to the SIR model (Susceptible Infectious Recovered Model), the urban traffic system in the epidemic times can be divided into five stages: peacetime stage, epidemic latent stage, epidemic outbreak stage, post-epidemic stage and recovery and upgrading stage [1]. By March, 2020, the rate of resumption of work in Shanghai, Jiangsu, Zhejiang, Fujian, Liaoning, Jiangxi, Guangdong and other provinces has exceeded 70%, and many places have started the initial stage to resume work and production. The Ministry of Transport of China has introduced measures such as strictly controlling the full load rate of public transport, lifting traffic restrictions and lowering parking rates to support economic activities while ensuring the safety of travelers [2, 3].

China has a huge population. The imbalance between the intercity passenger transport service level and the extremely high holiday travel demand is prominent. During the epidemic, intercity transport was greatly affected. In the post-epidemic stage, with the release of lock-down in some areas and the recovery of tourism and other service industries, this imbalance became more outstanding.

Most of the existing research results on travel behaviors are applicable to the pre-epidemic period, but there are few studies on the epidemic period and the post-epidemic times. The travel of residents under the influence of the epidemic is influenced by various factors (e.g., government control and their own psychological factors). Residents in cities with different levels of economic development have different perceptions of the travel risks associated with the epidemic, and the government’s management of residents’ travel needs to be considered based on social conditions (e.g., whether it is on a holiday), economic conditions, and the city’s geographic location. Traditional travel behavior research methods focus more on the activity travel itself, with less research on the interaction of the above-mentioned external factors, and also lack of in-depth discussion on the decision mechanism of travel behavior. Studying the intercity travel behaviors of residents in the post-epidemic times on holidays can not only provide decision-making basis for the planning, layout, design, traffic management and control of transportation infrastructure in the recovery and upgrading stage, but also help to restore people’s trust in public transport and improve its service quality [4].

Complex Network Analysis Theory and Evolutionary Game Theory are widely used in the research of transportation related fields. Yang et al. [5] used Complex Network Theory to evaluate the robustness of Beijing metro network in the face of random failures and malicious attacks. Ling et al. [6, 7] adopted Complex Network Theory to study the role of dynamic characteristics of traffic in dynamic networks and the traffic processes of static networks in explosive synchronization. Yu et al. [8] studied Nanjing metro network by using Complex Network Theory. Their study took metro lines as subsystems and further simplified them as nodes, providing perspectives for complex network research. Meng et al. [9] employed the Complex Network Theory to study the optimization of train timetable, and proposed practical methods to improve the stability of train timetable. Zhang et al. [10] analyzed the stability of urban public transport network based on the Complex Network Theory, and provided some valuable insights for future public transport network planning. Talarico et al. [11] established a multi-mode safe transportation model according to Evolutionary Game Theory. Based on this model, safety resources in chemical supply chain were allocated, and transportation modes with different safety characteristics were selected for different transportation scenarios. Li et al. [12] used the topology structure of the complex network to characterize the interaction between travelers. Based on the assumptions of travelers’ bounded rationality and crowd wisdom, an evolutionary game model of travelers’ travel was established and the travel behavior rules of travelers was studied during rush hours. Chen et al. [13] adopted evolutionary game theory to dynamically analyze the parking decision-making behaviors of government management departments, cargo transportation enterprises and freight drivers, so as to reduce the negative impact of unreasonable parking behaviors on the traffic system in the process of freight transportation.

Currently, scholars have conducted a series of studies on the travel intentions of tourists and the spatial and temporal characteristics of human activities during the COVID-19 epidemic. Li et al. [14] found that travelers significantly reduced the scope of intercity travel during the May Day holiday in 2020; Ye et al. [15] found that the risk level of the epidemic in Guangdong Province was largely influenced by the scale of population movement and transportation location factors; Wu et al. [16] found that the tourism market in Hong Kong’s outlying islands and Kowloon was most severely affected by the epidemic. The above studies suggest that the COVID-19 epidemic has a significant impact on the spatial and temporal patterns of human activities, leading to large fluctuations in the structure of travel networks.

Although relevant studies on the impact of the epidemic on residents’ intercity travel behavior have been conducted in the industry, they are mostly in the form of questionnaire surveys with limited sample size, which cannot reflect the changes in residents’ intercity travel patterns on a macroscopic scale. So far, few studies have been conducted on the travel behaviors combining Evolutionary Game Theory and Complex Network Analysis Theory. Evolutionary Game Theory and Complex Network Analysis Theory can both reflect the changes of residents’ travel patterns on a fine spatial and temporal scale and effectively describe the relationship between the government and residents in intercity travel activities. The intercity traffic network is a typical complex system, and the participants of intercity traffic, as a game group, cannot quickly select the optimal strategy every time. Therefore, based on traditional research on ways of traveling, the study adopted the Complex Network Analysis Theory. The city clusters of Shandong Peninsula were taken as the research region. A dynamic evolution model of how residents choose to travel was built to simulate the changes to their ways of traveling in the post-epidemic times under two conditions, which are: traveling under the government’s supervision of intercity travel and traveling under the government’s optimization of intercity travel conditions.

## 2. Location analysis of city clusters of Shandong Peninsula

### 2.1 Urban location analysis theory

There are various reasons for the heterogeneity of urban residents’ travel behaviors, including the differences in residents’ travel purpose, travel time and regional attributes [17]. In this section, the complex network method is adopted to analyze the urban network characteristics of city clusters of Shandong Peninsula.

The population migration network in the real world often features a small world and is scale free. The commonly used network analysis indicators are as follows:

(1) Degree. It is used to represent the number of edges connected to a node in a complex network. In a directed network, there are two concepts: in-degree and out-degree. Therefore, the population in-migration and out-migration intensity of any city in the study period can be expressed by Eqs (1) and (2):

$$W_{m\_i}=\sum_{j=1}^{n}R_{m\_ij}$$ (1)

Where *W*_*m_i*_ represents the in-migration intensity of city *m* in the study period, it is used to characterize the population migration scale per unit time. *R*_*m_ij*_ represents the value of the path where other cities have an inflow to city *m* within day *j*, and *n* represents the number of cities in a region.

$$W_{m\_o}=\sum_{j=1}^{n}R_{m\_oj}$$ (2)

Where *W*_*m_o*_ represents the migration intensity of city m in the study period (*o* represents out), and *R*_*m_oj*_ represents the value of the path where city *m* has an outflow to other cities within day *j*.

(2) In order to study the position potential of cities in the network, the weighted centrality index(*WCI*_*i*_) [18] and the city weighted advantage coefficient (*WAC*_*i*_) are used to calculate the position potential and advantage of cities in the network.

The index calculation is expressed by Eqs (3) and (4):

$$WCI_{i}=D_{i}^{\alpha }\times {\left(T_{i}/D_{i}\right)}^{\left(1-\alpha \right)}$$ (3)

Where *T_i_* is the sum of the inflow and outflow population of city *i*; *D_i_* is the sum of the in-migration and out-migration intensities of city *i*; α is the value assignment parameter, which is taken as 0.5; *WCI*_*i*_ represents the absolute position potential of city *i* in the network. The larger the value, the higher the absolute position potential level of city *i* in the whole network.

$$WAC_{i}=\frac{T_{i}}{\sum_{j=1}^{J}T_{j}/J}$$ (4)

Where *J* is the total number of cities in the network, and *i*≠*j*; *WAC*_*i*_ indicates the relative advantage of city *i*, which shows the level of relative advantage of each city in the whole intercity travel network. The greater the value, the stronger the relative advantage of city *i*. If *WAC*_*i*_ is greater than 1, it suggests that the advantage of the city is higher than the average level of the network.

(3) The urban equilibrium coefficient *UEC*_*c*_ is used to calculate the hierarchical structure characteristics of each city in the network. The calculation is shown in Eq (5):

$$UEC_{c}=-\sum_{i=1}^{I}\frac{Z_{i}\;\text{ln}\;Z_{i}}{\text{ln}(I-1)}$$ (5)

Where *Z_i_* represents the ratio of the sum of edge intensity associated with city *i* to the sum of edge intensity associated with all cities in the network. *I* represents the number of cities in the network. The value range of *UEC*_*i*_ is [0, 1]. When *UEC*_*c*_ = 0, it indicates that the difference of city level in the network is the largest. This index is used to describe the difference of city level of all cities in the whole intercity travel network.

(4) The ratio of the migration willingness index to the actual migration index from the Gaud migration big data is used to obtain the migration willingness, which characterizes the intercity migration willingness of the urban residents in the network. The calculation equation is as follows:

$$D_{\text{c}}=\frac{\sum_{\text{i}}^{m}\sum_{j}^{n}W_{ij}}{\sum_{\text{i}}^{m}\sum_{j}^{n}R_{ij}}$$ (6)

Where *m* is the time range (in days) of the study; *n* is the number of migration routes between cities in the region of the study; W_*ij*_ and R_*ij*_ represent the migration willingness index and the actual migration index.

### 2.2 Data acquisition

The urban network is usually studied by using direct data and indirect data based on population flow [19]. The direct data includes big data from Tencent location, Baidu migration data, and Gaud Map traffic big data. The indirect data includes train schedule data, passenger coach schedule data, and flight schedule data. In this study, big data from Gaud is used to show the willingness of urban migration. The in-migration intensity and out-migration intensity are used to characterize the intensity of population flow between cities in the areas of the study, so as to measure the interaction between cities in the areas. The intended migration data and actual migration data on weekdays and holidays before the epidemic (New Year’s Day holiday in 2019 and New Year’s Day holiday in 2020) are compared (see the data listed in Tables 1–8) with the holidays during the post-epidemic period (National Day holiday in 2021, New Year’s Day holiday in 2022 and the May Day holiday in 2022 respectively correspond to holiday 1 to 3 below) to quantitatively analyze the impact of the presence or absence of COVID-19 on the intercity travel willingness of urban residents in weekdays and holidays, in pre-epidemic and post-epidemic times, and during holidays. OD matrix A-F is generated by using the migration willingness index and the actual migration index among cities in the region of the study (where the letters A, B, C, E, F, G, K and L listed in Tables 1–8 represent the license plate letters of cities Jinan, Qingdao, Zibo, Dongying, Yantai, Weifang, Weihai and Rizhao, respectively).

**Table 1:** Migration willingness index and actual migration index of cities during the New Year’s Day holiday in 2019.

Date	City	Adcode	Willing out	Actual out	Willing in	Actual in
01–01	Jinan	370100	61.54	33.15	50.23	25.65
01–02			48.48	25.11	49.83	24.94
01–03			51.03	25.22	55.97	29.15
01–01	Qingdao	370200	37.01	17.96	30.22	13.70
01–02			31.41	13.63	31.41	14.59
01–03			51.03	25.22	34.53	16.99
01–01	Yantai	370600	16.13	7.38	17.56	8.79
01–02			15.76	7.03	15.83	7.38
01–03			16.76	7.65	16.15	7.44
01–01	Weihai	371000	6.15	2.52	7.75	3.40
01–02			6.35	2.60	6.88	2.78
01–03			6.46	2.67	6.82	2.65
01–01	Rizhao	371100	13.84	7.67	12.91	7.44
01–02			12.96	7.16	11.38	6.37
01–03			13.91	7.75	11.82	6.55
01–01	Dongying	370500	11.83	6.17	11.09	6.56
01–02			11.11	5.63	10.60	6.31
01–03			11.79	5.95	11.20	6.64
01–01	Weifang	370700	36.31	18.78	30.70	17.37
01–02			33.95	17.45	27.87	15.21
01–03			37.11	19.04	28.37	15.28
01–01	Zibo	370300	25.45	13.12	19.78	11.56
01–02			23.55	12.11	18.39	10.66
01–03			24.92	12.66	18.60	10.61

**Table 2:** Migration willingness index and actual migration index of cities during the New Year’s Day holiday in 2020.

Date	City	Adcode	Willing out	Actual out	Willing in	Actual in
01–01	Jinan	370100	23.24	11.63	24.59	12.30
01–02			21.71	10.05	22.97	10.64
01–03			22.38	10.82	23.68	11.45
01–01	Qingdao	370200	17.36	6.98	18.10	7.28
01–02			16.52	6.03	17.23	6.29
01–03			16.94	6.61	17.66	6.89
01–01	Yantai	370600	9.19	3.74	9.52	3.87
01–02			7.80	2.84	8.08	2.94
01–03			8.05	3.04	8.35	3.15
01–01	Weihai	371000	3.55	1.25	3.65	1.29
01–02			3.03	0.91	3.11	0.94
01–03			3.14	1.00	3.22	1.02
01–01	Rizhao	371100	7.30	3.91	7.45	3.99
01–02			6.25	3.10	6.38	3.16
01–03			6.34	3.29	6.47	3.36
01–01	Dongying	370500	6.94	3.41	7.08	3.48
01–02			6.13	2.94	6.25	3.00
01–03			6.76	3.33	6.89	3.40
01–01	Weifang	370700	19.51	9.67	20.11	9.97
01–02			16.48	7.73	16.99	7.98
01–03			16.81	8.26	17.33	8.52
01–01	Zibo	370300	13.12	6.45	13.53	6.65
01–02			11.20	5.29	11.55	5.46
01–03			11.48	5.71	11.83	5.89

**Table 3:** Matrix A—Intercity migration willingness index of city clusters of Shandong Peninsula during the National Day holiday in 2021.

	A	B	C	E	F	G	K	L
A	0	7.21	11.12	3.03	5.87	8.85	2.91	3.83
B	5.95	0	3.52	1.72	17.5	18.04	6.98	8.19
C	11.8	4.83	0	3.45	3.52	11.48	2.07	1.88
E	2.64	2.4	2.48	0	2.18	5.69	1.01	0.56
F	2.38	9.25	1.17	0.87	0	4.12	9.78	1.01
G	8.18	20.13	8.41	5.42	9.51	0	3.9	7.48
K	0.83	2.28	0.43	0.24	5.52	1.02	0	0.31
L	1.58	7.31	0.62	0.29	1.46	3.93	0.87	0

**Table 4:** Matrix B—Intercity actual migration index of city clusters of Shandong Peninsula during the National Day holiday in 2021.

	A	B	C	E	F	G	K	L
A	0	2.38	5.25	1.3	2.19	3.98	0.97	1.44
B	1.92	0	1.5	0.96	8.57	9.24	3.32	4.11
C	5.2	1.73	0	1.48	1.42	4.92	0.85	0.71
E	0.99	1.03	1.23	0	0.98	2.87	0.44	0.23
F	0.66	4.3	0.48	0.31	0	1.97	4.74	0.38
G	3.26	9.35	4.45	2.85	4.67	0	1.89	3.28
K	0.2	0.81	0.15	0.06	2.72	0.41	0	0.1
L	0.46	3.15	0.25	0.11	0.61	2.06	0.36	0

**Table 5:** Matrix C—Intercity migration willingness index of city clusters of Shandong Peninsula during the New Year’s Day holiday in 2022.

	A	B	C	E	F	G	K	L
A	0	1.62	5.47	1.25	0.84	3.17	0.29	0.64
B	1.59	0	1.02	0.57	7.4	8.6	1.61	2.68
C	5.22	1.14	0	1.63	0.49	5.08	0.17	0.38
E	1.03	0.63	1.19	0	0.32	2.47	0.09	0.14
F	0.66	5.02	0.3	0.24	0	1.59	3.43	0.24
G	2.74	8.94	3.76	2.81	2.35	0	0.48	2.4
K	0.21	0.91	0.08	0.06	2.65	0.26	0	0.07
L	0.52	2.72	0.23	0.15	0.36	1.81	0.13	0

**Table 6:** Matrix D—Intercity actual migration index of city clusters of Shandong Peninsula during the New Year’s Day holiday in 2022.

	A	B	C	E	F	G	K	L
A	0	0.63	3.04	0.66	0.31	1.7	0.08	0.27
B	0.52	0	0.5	0.28	4.42	5.39	0.83	1.65
C	2.7	0.46	0	0.86	0.2	2.43	0.05	0.15
E	0.44	0.28	0.7	0	0.14	1.39	0.03	0.07
F	0.19	2.72	0.14	0.11	0	0.87	2.01	0.09
G	1.23	4.89	2.21	1.69	1.27	0	0.21	1.27
K	0.04	0.38	0.02	0.02	1.56	0.11	0	0.03
L	0.19	1.44	0.1	0.07	0.17	1.1	0.05	0

**Table 7:** Matrix E—Intercity migration willingness index of city clusters of Shandong Peninsula during the May Day holiday in 2022.

	A	B	C	E	F	G	K	L
A	0	0.92	1.59	0.31	0.35	0.91	0.17	0.29
B	0.85	0	0.82	0.42	2.84	5.65	1.18	2.4
C	1.36	0.98	0	0.83	0.23	2.92	0.15	0.24
E	0.26	0.53	0.71	0	0.14	1.32	0.08	0.12
F	0.24	2.2	0.14	0.1	0	0.6	1.1	0.13
G	0.81	5.91	2.28	1.42	0.85	0	0.39	1.56
K	0.1	0.74	0.08	0.05	0.74	0.23	0	0.07
L	0.22	2.33	0.21	0.11	0.21	1.34	0.14	0

**Table 8:** Matrix F—Intercity actual migration index of city clusters of Shandong Peninsula during the May Day holiday in 2022.

	A	B	C	E	F	G	K	L
A	0	0.28	0.71	0.13	0.08	0.32	0.03	0.08
B	0.21	0	0.36	0.2	1.42	3.14	0.57	1.37
C	0.55	0.39	0	0.4	0.08	1.65	0.05	0.1
E	0.07	0.23	0.34	0	0.05	0.67	0.03	0.05
F	0.04	1.02	0.05	0.03	0	0.2	0.45	0.05
G	0.27	3.05	1.22	0.79	0.35	0	0.17	0.72
K	0.01	0.3	0.03	0.01	0.3	0.08	0	0.03
L	0.06	1.28	0.1	0.05	0.1	0.66	0.07	0

### 2.3 Analyses of calculation results

The ratio of the migration willingness index to the actual migration index of the three holidays was calculated to characterize the intercity migration willingness of the residents in all cities of the network. See the data in Table 9 for the results.

**Table 9:** Calculation results of migration willingness.

Time	Pre-epidemic weekdays	Pre-epidemic holidays	Holiday 1	Holiday 2	Holiday 3
D_c_	0.49	0.46	0.37	0.40	0.35

The weighted centrality index *WCI*_*i*_ of each city in the three holidays (holiday 1 to 3) is calculated respectively, which is compared with that of the weekdays and holidays of eastern cities before the epidemic (Table 10) [14]. The results are shown in Table 11. The *UEC*_*c*_ of city clusters of Shandong Peninsula is shown in Table 12.

**Table 10:** Average *WCI*_*i*_ of weekdays and holidays before epidemic.

	The whole country		East	
Time	Weekdays	Holidays	Weekdays	Holidays
*WCI*_*i*_ mean	18.52	38.67	30.5	58.12

**Table 11:** *WCI*_*i*_ of city clusters of Shandong Peninsula during three holidays after epidemic.

	Holiday 1	Holiday 2	Holiday 3
Jinan	30.2	12	2.84
Qingdao	52.37	24.39	13.82
Zibo	29.62	13.56	6.03
Dongying	14.84	6.74	3.05
Yantai	34	14.2	4.22
Weifang	55.2	25.76	13.29
Weihai	17.02	5.42	2.13
Rizhao	17.25	6.65	4.72

**Table 12:** Urban equilibrium coefficient of city clusters of Shandong Peninsula.

Time	*UEC*_*c*_
Holiday 1	1
Holiday 2	0.99
Holiday 3	0.95

The *WAC*_*i*_ of each city in Shandong Peninsula was calculated. The calculation results are shown in Table 13 (*the specially marked value indicates that the advantage value of the city is higher than that of the average level of cities in network*).

**Table 13:** Weighted advantage coefficient *WAC*_*i*_ of each city.

	Holiday 1	Holiday 2	Holiday 3
Jinan	0.96	0.88	0.45
Qingdao	1.67	1.79	2.21
Zibo	0.95	1.00	0.96
Dongying	0.47	0.50	0.49
Yantai	1.09	1.04	0.67
Weifang	1.76	1.90	2.12
Weihai	0.54	0.40	0.34
Rizhao	0.55	0.49	0.75

The roles of cities in Shandong Peninsula were divided according to the urban role identification model [20]. The results are shown in Table 14.

**Table 14:** Roles of cities.

	Holiday 1	Holiday 2	Holiday 3
Regional hub city	Weifang, Qingdao	Weifang, Qingdao	Qingdao, Weifang
Local hub city	Yantai, Jinan, Zibo	Yantai, Zibo, Jinan	—
Normal city	Rizhao, Weihai, Dongying	Rizhao, Dongying, Weihai	Zibo, Yantai
Edge city	—	—	Dongying, Jinan, Weihai

According to the data in Table 9, the willingness of residents to migrate on short-term holidays is higher than that on long-term holidays, and the willingness to migrate on holidays is generally lower than that before the epidemic. According to the results of urban equilibrium coefficient of city clusters of Shandong Peninsula in Table 12, this value is very close to 1 in all three holidays, which shows that there is no obvious difference in the city level of the whole intercity travel network. Before and after the holiday 1 (National Day holiday in 2021), there were no local COVID cases in Shandong Province; the travel of residents was less restricted, and was therefore normal. Moreover, the duration of the National Day holiday was long. Therefore, Shandong Peninsula saw the largest intercity population flow on holiday 1. The weighted centrality index of Qingdao and Weifang, the regional hub cities in Shandong Peninsula city clusters, is also the closest to the average value of eastern cities during the National Day holiday before the epidemic. As the capital city of Shandong Province, Jinan’s relative position potential is not as good as Weifang and Qingdao. First, the intercity travel in this study is only limited to the city clusters of Shandong Peninsula, and does not involve other cities outside the region. Second, Qingdao and Weifang are located in the center of the region, which have strong attraction to the surrounding cities in the region. Before and after the holiday 2 (New Year’s Day holiday in 2022), there were no local COVID cases in Shandong Province, while cases of Omicron, which was highly infectious, occurred in some parts of China. The travel of residents in Shandong Peninsula was less restricted, and was therefore basically normal. The external environment of intercity travel was basically the same as that of holiday 1. The roles of cities in the region were roughly the same as those of holiday 1. The duration of New Year’s Day holiday was short, thus the intensity of residents’ migration during this period is low. However, the willingness of residents’ migration is 0.40, which is slightly higher than 0.37 of holiday 1. This indicates that the intercity traffic management capacity of Shandong Peninsula has been improved, and that the trust among intercity traffic was recovering in an orderly manner. Before the holiday 3 (the May Day holiday in 2022), there were concentrated Omicron cases in many places in Shandong Province. Shandong Provincial Health Commission designated 86 lock-down areas, 130 control areas, 67 prevention areas in Jinan. It designated 150 lock-down areas and 60 control areas in Yantai. Strict measures were taken against the epidemic. There were many travel restrictions for residents in Shandong Peninsula, and some urban public transport has been suspended. The epidemic has directly led to a significant reduction in the connection between the two cities and other cities. These two cites have a high position potential in Shandong Peninsula. As a result, this has further affected the willingness of all urban residents in the region to travel between cities.

## 3. Ways of travel selection model

### 3.1 Evolutionary game analysis

The single OD pair traveling by two ways (public transport and private transport) is considered. Assume that the total traffic demand is N and that the public transport supply can fully meet the traffic demand. The travel method selection problem between the OD pair can be regarded as a group game problem, and the game elements are as follows:

(1) Let the selection set of the two travel modes by travelers between the OD pair be S = {*s*_*1*_, *s*_*2*_}.
(2) The proportion of travelers choosing public transport is *x*, and that choosing private transport is *(1-x)*.
(3) Assume that the travel cost is *c*_*i*_ when the traveler selects *s*_*i*_, hence the travel benefit is the inverse of the travel cost -*c*_*i*_ when the traveler selects *s*_*i*_.
(4) In the case of road congestion, the cost of choosing private transportation is c_1_, the additional travel cost caused by road congestion is c_3_, and when both sides of the game use private transportation, the travel cost of both sides of the game is c_1_+c_3_; When the game opponent chooses public transportation, it will not cause road congestion, and the travel cost of private transportation is c_1_; The price and travel time of public transportation are relatively certain, so no matter what kind of travel method the other party chooses, the travel cost of the traveler choosing public transportation is c_2_.

Based on the above, the cost matrix of travel mode selection is obtained (see Table 15).

**Table 15:** Cost matrix of travel mode selection.

Ways of Travel	Private Transport	Public Transport
Private transport	(c_1_+c_3_,c_1_+c_3_)	(c_1_,c_2_)
Public transport	(c_2_,c_1_)	(c_2_,c_2_)

According to the above and from Eqs (7) and (8), the expected benefits of travelers choosing private transport and public transport can be obtained, as shown in the following:

$$F_{1}=-(c_{1}+c_{3})x-c_{1}(1-x)$$ (7)

$$F_{2}=-c_{2}x-c_{2}(1-x)=-c_{2}$$ (8)

Where *F*_*1*_ is the benefit function of travelers choosing private transport, and *F*_*2*_ is the benefit function of travelers choosing public transport.

In the evolutionary game theory, the dynamic evolution equation is used to describe the changing speed of the proportion of strategy selection between the two sides of the game. The evolution dynamics can be divided into deterministic dynamics and stochastic dynamics. Among them, the deterministic evolution dynamics is expressed by the average dynamic equation, and the change rate of travel mode selection probability is used to describe the change law of travel mode selection of travelers. The rate of selection change probability is as follows:

$${\bar{x}}_{i}=\sum x_{j}\rho_{ji}-\sum x_{i}\rho_{ij}$$ (9)

Where *x*_*i*_ is the probability that the traveler selects the travel mode *i*; *ρ*_*ij*_ is the probability that the traveler shifts from mode *i* to mode *j*.

The conditional transition probability is as follows:

$$\rho_{ij}=\frac{e^{Fi}}{\sum_{k\in S}e^{Fk}}$$ (10)

The Logit dynamic evolution equation is obtained by substituting Eq (10) into Eq (9), as shown in Eq (11):

$${\bar{x}}_{i}=\frac{e^{Fi}}{\sum_{k\in S}e^{Fk}}-x_{i}$$ (11)

Where *F*_*i*_ is the expected benefit function of a traveler’s target travel mode *i*; *F*_*k*_ is the expected benefit function when a traveler chooses travel mode *k*; *S* represents the strategy set of two travel modes selected by travelers between OD pairs.

The Logit dynamic model of travelers’ travel mode selection is obtained by combining Eqs (7), (8) and (11), and the change rate of travelers choosing private transport is:

$$\bar{x}=\frac{1}{1+e^{A_{x}+B}}-x$$ (12)

Where *A* = *c*_*3*_ ≥ 0 indicates the additional travel cost caused by road congestion; *B* = *c*_*1*_* − c*_*2*_ means the difference between the cost of private transport and public transportation when the expressway is not congested, which in actual situations represents the inherent cost difference between private transport and public transport.

Let the above equation be equal to 0, and the following is obtained:

$$x=\frac{1}{1+e^{A_{x}+B}}$$ (13)

Let

$$y=A_{x}+B$$ (14)

Substitute Eq (14) into Eq (13) to obtain the following:

$${\text{e}}^{y}=\frac{1}{x}-1$$ (15)

Apply logarithm to the equations to obtain the following:

$$y=\text{ln}\;\left(\frac{1}{x}-1\right),\;x\neq 0$$ (16)

Combine Eqs (14) and (16). As *A* is greater than 0, there is a unique solution to this equation system, and the obtained equilibrium point is shown in Fig 1.

**Fig 1:** Equilibrium diagram.

The influence of the change of parameters *A* and *B* in Eq (13) on the equilibrium point x* is analyzed as follows:

If the value of *A* becomes larger, causing the equilibrium point *x* * to shift to the left, it means that the cost difference between road congestion and non-congestion increases when travelers choose private transport, that is, the delay cost of choosing private transport increases. According to the principle of maximum utility, some travelers who choose private transport will change their travel mode. If the value of *B* becomes large, causing the equilibrium point x* to shift to the left, it means that the difference between the travel cost of private transport and public transport increases when the road is not congested. Some travelers who choose private transport will change their travel mode. If the value of *A* decreases, causing the equilibrium point *x* * to shift to the right, it means that the cost difference between road congestion and non-congestion decreases when travelers choose private transport. The model becomes stable. If the value of *B* decreases, causing the equilibrium point x* to shift to the right, it means that the difference between the travel cost of private transport and public transport reduces when the road is not congested. The model becomes stable.

To sum up, if the government plans to increase the proportion of public transport trips, a number of measures need to be taken to make the equilibrium point of this model shift to the right. In the model, parameter *A* actually represents the delay cost whether the road is congested or not, and parameter *B* actually represents the difference in time cost and economic cost caused by the inherent attributes of private transport and public transport. Therefore, the residents can be encouraged to choose public transport during intercity travel by increasing the frequency of intercity railway trains and their speed, opening express lines of intercity railway trains in big stations, reducing the ticket price, and changing the expressway tolling mode (e.g., tolls can be based on both time and mileage).

### 3.2 Numerical simulation and calculation

To more intuitively show the trend of private and public transport travel affected by policies, the above model is numerically simulated and calculated. Assume that expressway tolls are exempted on holidays, the travel cost of private transport between an OD pair comes from fuel cost and time cost, and the travel cost of public transport comes from ticket price and time cost [21], thus there is the following:

$$c_{i}=t_{i}+\frac{m_{i}}{\gamma }$$ (17)

Where *c*_*i*_ is the time cost for residents to choose travel mode *i*, and *m*_*i*_ is the fuel cost or ticket price; γ is the unit time cost, which is assumed to be 20 (yuan / hour) in the calculation in this section.

(1) The most representative OD pair is analyzed, which is Jinan-Qingdao pair in the studied region. Assume the proportion of group 1 choosing private transport is *x*, and that choosing public transport is (*1-x*); the proportion of group 2 choosing private transport is *y*, and that choosing public transport is (*1-y*). The expressway is about 360 kilometers long, and the traffic time is about 4 hours if there is no congestion and 6 hours if there is congestion. The economic cost is assumed to be 200 yuan. Therefore, there are the following equations: *c*_*1*_ = 4 + 200/20 = 14*h*, *c*_*1*_*+c*_*3*_ = 6 + 200/20 = 16*h*; For public transport, intercity coaches and trains are considered comprehensively: *c*_*2*_ = 4 + 140/20 = 11*h*. Based on the above conditions, the cost matrix of this OD pair for travel mode selection is given below (Table 16). The evolution game process of travel mode selection is shown in Fig 2(a).

**Fig 2:** Evolution game process of travel mode selection behaviors.

**Table 16:** Cost matrix of travel mode selection.

Ways of Travel	Private transport	Public transport
Private transport	(16,16)	(14,11)
Public transport	(11,14)	(11,11)

The following is an analysis of the dynamic evolution process of residents’ travel behavior under the government’s involvement and supervision after a local small-scale epidemic occurs in a period such as holiday 3. The government’s supervision on intercity travel is mainly to restrict the full load rate of public transport and impose on procedures for residents to enter and leave the bus station and railway station. In the model, this indicates the increase of the time cost of public transport. Then there is the equation: *c*_*2*_ = 5 + 140/15 = 14.33*h*, and this situation is shown in Fig 2(b).

According to Fig 2(a), this evolutionary game process tends to be stable after a limited number of iterations. It indicates that the residents’ intercity travel mode selection behavior between Jinan and Qingdao tends to be stable. Therefore, the proportion of residents choosing public transport will increase with the gradual restoration of residents’ trust in public transport. Under the government’s involvement and supervision, as shown in Fig 2(b), public transport no longer dominates the modes of travel between the two places. If the government wants to restore the dominant position of public transport under this condition, it can introduce measures such as simplifying the entry and exit procedures and properly increasing the full load rate on the premise of ensuring the safety of passengers.

(2) For the travel between two cities with little difference in position potential in a short distance, the OD pair of Zibo and Weifang is analyzed. The expressway is about 120 kilometers long, and the traffic time is about 1.5 hours if there is no congestion and 2.5 hours if there is congestion. The economic cost is assumed to be 50 yuan. Therefore, there are the following equations: *c*_*1*_+*c*_*3*_ = 2.5 + 50/20 = 5*h*; *c*_*1*_ = 1.5 + 50/20 = 4*h*. For public transport, intercity coaches and trains are considered comprehensively: *c*_*2*_ = 1.5 + +60/20 = 4.5*h*. Based on the above conditions, the cost matrix of this OD pair for travel mode selection is given below (Table 17).

**Table 17:** Cost matrix of travel mode selection.

Ways of Travel	Private Transport	Public Transport
Private transport	(5, 5)	(4, 4.5)
Public transport	(4.5, 4)	(4.5, 4.5)

Under the condition that the public transport is optimized by adjusting the travel time cost to 4h (in reality, this can be realized by reducing the ticket price by 10 yuan), output the dynamic evolution process of residents’ travel behavior under the government’s involvement and supervision after a local small-scale epidemic which occurs during holiday 3. See Fig 3.

**Fig 3:** Evolution game process of travel mode selection behaviors.

According to Fig 3(a), the evolutionary game process of travel mode selection behavior between Weifang and Zibo will not be stable after a limited number of iterations, and under the existing conditions, residents are more inclined to choose private transport. If public transport is optimized by adjusting the travel time cost to 4h (in reality, this can be realized by reducing the ticket price by 10 yuan), as shown in Fig 3(b), although the evolutionary game process is still not stable, the proportion of residents choosing public transport for travel increases significantly. As the fixed cost determined by the inherent nature of public transport cannot be reduced, the parameters in this case will not be adjusted. If government’s supervision is considered, as shown in Fig 3(c), this evolutionary game process tends to be stable after a limited number of iterations. This indicates that residents’ intercity travel mode selection behavior between Weifang and Zibo tends to be stable, and that residents are more willing to choose private transport.

## 4. Discussions

(1) The data obtained in this study suggest that the locational relationships among cities in urban agglomerations may change due to the impact of the epidemic, and the roles of cities in urban agglomerations may change in response to changes in the epidemic situation and government policies on epidemic prevention.
(2) Changes in city roles and urban locations can change the extent to which the epidemic affects residents’ intercity travel choice behavior. In the city cluster of Shandong Peninsula selected for this study, travel between the two hub cities Jinan-Qingdao is dominated by public transportation in general, but under the influence of the epidemic and government involvement in regulation, residents’ trust in public transportation will decrease, and some residents will prefer private transportation for travel. In trips between two cities with short distances and little difference in location, Zibo-Weifang, residents always tend to choose private transportation trips unless the government intends to optimize public transportation trips.
(3) At present, travel during holidays is still significantly affected by the epidemic. Before and after the National Day holiday in 2021 and the New Year’s Day holiday in 2022, the travel situation of residents was not so different from that during the holidays before the epidemic. This situation to a certain extent reflects the improvement of the management capacity of intercity traffic in Shandong Peninsula and the continuous enhancement of the “certainty” for residents to travel. The trust among intercity traffic is recovering in an orderly manner. However, before the May Day holiday in 2022, there were concentrated Omicron cases in many places in Shandong. There were many travel restrictions for residents in Shandong Peninsula, and some urban public transport has been suspended.
(4) The limitations of this paper are mainly reflected in the following two aspects. On the one hand, due to time constraints, the study of residents’ travel behavior during holidays in the post-epidemic era only covers some holidays in the past two years, and there are problems such as incomplete data collection and small samples; on the other hand, the study of intercity travel in this paper is only limited to the inner city cluster, and does not consider the connection between cities within the city cluster and cities outside the region.
(5) Future studies need to collect more extensive and comprehensive data, and take into account other factors influencing travel behavior, for example, adding consideration of latent variables such as residents’ perceived risk capacity, economic constraints, and travel time.

## 5. Conclusion

(1) On the whole, the neighboring cities in Shandong Peninsula are closely connected, and the intercity travel is dominantly between neighboring cities. The migration intensity between Yantai and Weihai, Weifang and Qingdao, and Jinan and Zibo is prominent. The strong attraction between neighboring cities also leads to the weak overall connection of the urban network in Shandong Peninsula. The provincial capital city Jinan and the sub-provincial city Qingdao have limited attraction to non-neighboring cities in the region, and there is no obvious difference in the city level of the whole intercity travel network.
(2) According to the current data, the travel network concentration of residents in long-term holidays is lower than that in short-term holidays, and the migration intensity of residents is higher than that in short-term holidays, while the willingness of resident migration in short-term holidays is higher than that in long-term holidays. The willingness to migrate during the holidays is lower than that before the epidemic. For one thing, this suggests that the travel willingness of residents in the post-epidemic era is still recovering. For another, this shows that the intercity traffic management capacity in the post-epidemic era needs to be improved, and that the recovery and development of the traffic field are still complex.
(3) The epidemic has directly led to a significant reduction in the connection between the two cities and other cities. These two cites have a high position potential in Shandong Peninsula. As a result, this has further affected the willingness of all urban residents in the region to travel between cities. Besides, the epidemic will affect the change of the equilibrium coefficient of the city clusters, which lead to a more significant city level difference among the cities in the network. For example, in the region of the study, the urban advantage of Qingdao and Weifang is significantly higher than that of other cities due to the epidemic.
(4) In the intercity travel network, the travel between two cities with medium and long distances is normally dominated by public transport. Due to the impact of COVID-19, the dominant position of public transport will be affected, but it will not be replaced by private transport. In short-distance travel between two cities, private transport is in an advantageous position, and under the impact of the epidemic, this position will become dominant. The government can improve the position of public transport in short-distance travel by making optimizations (such as appropriately reducing ticket prices and simplifying entry and exit procedures).
(5) There are many kinds of direct linked data and indirect linked data in process of the study about intercity travel behavior during holidays, and the amount of data is large, which requires more powerful computing power. At the same time, in order to prevent some sensitive data information from being stolen by malicious attackers, federated learning model can be used to analyze and process traffic travel data, which is helpful to achieve better research results and ensure data security.

## Supporting information

S1 Appendix (DOCX)

S1 File (XLS)
